# Health Effects of Probiotics on Nonalcoholic Fatty Liver in the Life Cycle Based on Data Analysis

**DOI:** 10.1155/2022/2123162

**Published:** 2022-07-29

**Authors:** Jia Wang, Yanfei Hao, Xiao Jin, Xiaoyue Li, Yi Liu, Li Zhang, Jing Wang, Mingxin Hu

**Affiliations:** ^1^Department of Health Management, Aerospace Center Hospital, Beijing 10089, China; ^2^China Aerospace Academy of Systems Science and Engineering, Beijing 100037, China

## Abstract

**Objective:**

To observe the effect of intestinal probiotics in the treatment of nonalcoholic fatty liver disease (NAFLD) and the effect on liver function and inflammatory factors.

**Methods:**

34 healthy rats were selected for the study and divided into 10 rats in the control group, 12 rats in the model group, and 12 rats in the treatment group according to the random number table method. The control group was given behavioral and lifestyle interventions, and the treatment group was given Bifidobacterium minus Black enteric capsules 5 g/(kg-d) by strong feeding method on the basis of the control group. The fatty liver index (FLI), liver ultrasound examination results, liver function, and inflammatory factor levels were compared among the three groups. After 8 weeks of treatment, there were statistically significant differences between the FLI values and liver ultrasound results of the three groups, and the serum alanine aminotransferase (ALT), aspartate aminotransferase (AST), triacylglycerol (TG), and total cholesterol (TC) levels of the observation group were lower than those of the control group and the model group. The levels of serum high molecular weight lipocalin (HMW-APN) and interleukin 22 (IL-22) in the observation group were higher than those in the control group, and the levels of tumor necrosis factor-*α* (TNF-*α*) were lower than those in the control and model groups, and the differences were statistically significant (*P* < 0.05).

**Conclusion:**

Intestinal probiotics can improve the clinical efficacy of patients with NAFLD, improve liver function, and alleviate the inflammatory response, in order to provide a theoretical basis for the clinical treatment of patients with NAFLD.

## 1. Introduction

NAFLD is a clinicopathological syndrome characterized by diffuse hepatocellular steatosis, excluding alcohol and other definite hepatoprotective factors, and is classified into simple fatty liver, NAFLD, and associated cirrhosis based on the presence of inflammation and fibrosis [1]. The prevalence of NAFLD is as high as 57% and 98% in overweight and obese populations, respectively [2], and in recent years, as overweight and obesity rates in the Chinese population and obesity rates have been rising, the prevalence of NAFLD has been increasing rapidly and at a younger age.

The pathogenesis of NAFLD is currently considered to be the hepatic manifestation of the metabolic syndrome and has not been fully elucidated, but recent studies have shown that its development is closely related to changes in the intestinal flora and that disturbances in the intestinal flora and increased intestinal wall permeability play an important role in the development of NAFLD, mediated by an immune response [3]. Probiotics, represented by Lactobacillus and Bifidobacterium, have been shown to be directly associated with cholesterol metabolism, gastrointestinal infections, and bacterial translocation [4]. The use of probiotic preparations in NAFLD is currently uncommon, and the therapeutic effects and mechanisms of NAFLD are unknown [5]. In addition, common pharmacological treatments include vitamin E, pioglitazone, metformin, capsaicin, cloacenamide, and statins, of which the most effective pharmacological treatment is uncertain [6].

The pathogenesis of NAFLD is not fully understood. Recent theories suggest that because simple steatosis is a benign process in many patients, whereas NASH is a progressive process, NASH may have a unique pathogenesis in which the liver is exposed to a combination of insulin resistance, oxidative stress, enteric-derived endotoxins, bacterial endotoxins, altered adipocytosine profile, and reduced bile secretion, leading to an inflammatory response [7]. The traditional “second strike” theory suggests that the first strike, including hepatic fat accumulation and insulin resistance, leads to hepatic steatosis, which increases the release of inflammatory factors, adipocytosine, oxidative stress, and mitochondrial dysfunction (second strike) and ultimately leads to NASH and even liver fibrosis [8].

The human intestinal flora contains more than 1000 species of bacteria with a total of 1 × 1014 species, a mass of 1-2 kg, and a total number of genes exceeding 150 times the total number of host genes [9]. The intestinal flora may be influenced by multiple factors such as diet, lifestyle, age, host genotype, and drug use and is a dynamic combination of quantitative and species changes [10]. According to reports, increased intestinal mucosal permeability and SIBO are common in patients with NAFLD and correlate with the severity of hepatic steatosis [11]. Studies have shown that the bacterial endotoxin lipopolysaccharide (LPS) is hepatotoxic, is increased in the plasma of patients with diabetes, metabolic syndrome, and NAFLD, and plays an important role in the progression of NASH [12]. In addition, ecological dysbiosis of the intestinal flora can lead to an increase in bacterial synthesis of endogenous alcohol, resulting in the production of large amounts of reactive oxygen species during alcohol metabolism, which further increases intestinal mucosal permeability and promotes liver inflammation [13].

Nonalcoholic fatty liver disease (NAFLD) is a metabolic disease characterized by diffuse steatosis of hepatocytes, except for excessive alcohol consumption or other diseases based on fatty degeneration of hepatic parenchymal cells, which can progress to steatohepatitis, cirrhosis, and liver cancer [14]. The pathogenesis of NAFLD is still unclear, but it is currently considered to be related to lipid metabolism, insulin resistance, and inflammatory factor release, and it has been found that the “enterohepatic axis” of intestinal flora plays an important role in its pathogenesis. On the other hand, the endotoxin produced by the flora can cause high expression of inflammatory factors, which can lead to liver damage [15]. We used probiotics in the treatment of NAFLD in mice and observed the effect of intestinal probiotics on the treatment of NAFLD and the effect on liver function and inflammatory factors, in order to provide reference for clinical treatment.

## 2. Materials and Methods

### 2.1. Animals

We used 34 SD male rats (Beijing Weitong Lihua Laboratory Animal Technology Co., Ltd.), SPF grade, production license number SCXK (Zhejiang, China) 2016-0006, age about 8 weeks, weight about 300 g. TNF, IL-6 radioimmunoassay kits were provided by Wuhan Dr. Biotechnology Co. Basic feed formulation is as follows: 35% standard meal, 15.5% bran, 20% soybean meal, 20% corn meal, 0.5% soybean oil, 5% fish meal, 2.5% bone meal, and 1% yeast; high-fat feed formulation is as follows: 60% basal feed, 15% cooked lard, 10% egg yolk powder, 8% skim milk powder, 5% casein, and 2% white sugar. Japan Hitachi U2200 double-beam spectrophotometer, 7170 automatic biochemical analyzer, vortex mixer, low-temperature high-speed centrifuge, and Olympus IX71 inverted microscope were used. The animal room environment and cages were kept clean during the experimental period. During the experimental period, animals were provided with humane care according to the “3R” principle. The study was approved by the Animal Ethics Committee.

### 2.2. Methods

#### 2.2.1. Drug Interventions

Thirty-four rats were divided into 3 groups, 10 in the control group, 12 in the model group, and 12 in the treatment group, and continued to be fed a high-fat diet. The control group continued to be fed a basal diet. The treatment group was given Lactobacillus bifidum triple solution (4 tablets mixed with 20 mL distilled water) 5 g/(kg-d), 1 time/d by the strong feeding method, and 1 time/d; the same volume of saline was given to the model group by the strong feeding method. At the end of week 16, at 8 weeks, healthy subjects were performed and blood was collected for testing.

#### 2.2.2. Collection and Processing of Specimens

At the end of 8 weeks of dosing, rats are fasted for 12 hours. The abdominal cavity is rapidly opened, and blood is drawn from the abdominal aorta at 12,000 r/min. The serum is isolated and stored at -80°C to detect adipokines, lipids, and liver function. The rest of the liver is immediately frozen in liquid nitrogen and transferred to -80°C for freezing and storage.

#### 2.2.3. Indicator Testing

The liver index was calculated by weighing the wet mass of the liver and the body mass of the liver, and the liver/body ratio was calculated as the liver index. The fasting blood-glucose (FBG) was measured by a fully automated biochemical analyzer. Fasting insulin (FNS) was determined by the immunoassay method, and the insulin resistance index (HOMA-IR) was calculated as FPG × F N S/22.5. TNF-*α*, lipocalin, and IL-6 were determined by ELISA. Each section was examined under light microscopy for 5 × 400 fields of view to grade the degree of hepatic steatosis and inflammatory cell infiltration. The diagnosis was made by an experienced pathology faculty member who read the slides blindly.

Statistical analysis data were described as mean ± SD. The SPSS 16.0 statistical software was used for analysis, *t*-test was used for comparison between two groups, and one-way ANOVA was used for comparison between groups, and *P* < 0.05 was considered statistically significant.

## 3. Results

### 3.1. Comparison of Blood Lipids, Liver Function, and Liver Index

Serum triglycerides (TGs), total cholesterol (TC), alanine aminotransferase (ALT) and aspartate aminotransferase (AST), and liver index were significantly higher in the model group rats compared with the normal control group (*P* < 0.01); compared with the model group, TG, transaminases, and liver index were significantly lower in the treated group rats (*P* < 0.05); however, compared with the normal control group, they remained elevated (*P* < 0.05); TC levels in the treated group were not significantly reduced compared with the model group (*P* > 0.05, Table 1).

### 3.2. Changes in Liver Pathology in All Groups of Rats

The hepatocytes were radially distributed around the central vein without lipid infiltration, and there was no inflammatory cell infiltration in the confluent area and lobules (Figure 1(a)). In the NAFLD model group, the hepatocytes were disorganized and sparse, with poorly defined borders. Inflammatory cells were mainly lymphocytes (Figures 1(b) and 2(b)), which were significantly different from the normal control group (*P* < 0.01). Compared with the control group, steatosis was still present in the treated group, and the hepatocytes were sparsely arranged; however, the lipid droplets were smaller and more restricted, and the number of inflammatory cells infiltrating the confluent area was significantly lower compared with the model group (*P* < 0.01, Figures 1(c) and 2(c)).

### 3.3. Comparison of Serum Inflammatory Factors and Insulin Resistance in Rats

At the end of 16 weeks, serum IL-6, TNF-*α*, and HOMA-IR levels were significantly higher in the model group than in the normal control group, while lipocytin levels were significantly lower (*P* < 0.01). After 8 weeks of probiotic treatment, serum HOMA-IR, IL-6, and TNF-*α* levels decreased significantly (*P* < 0.05), while lipocytin levels increased but did not return to normal serum levels (*P* > 0.05, Table 2).

## 4. Discussion

In recent years, the incidence of NAFLD in China has been increasing year by year with the improvement of living standards. There is no definite mechanism for the pathogenesis of NAFLD, but the “second strike” theory, which is based on insulin resistance and lipid oxidative stress, has been widely accepted in previous studies [16]. However, this theory is still controversial. Based on anatomical and functional correlations, the concept of the “intestine-liver axis” suggests that the liver and intestine interact in multiple ways to provide for each other's immune integrity [17]. The role of intestinal barrier function in the pathogenesis of NAFLD is becoming an important aspect of research. The intestinal mucosal barrier is the sum of the structures and functions of the intestine that prevent harmful substances such as bacteria and toxins in the intestinal lumen from crossing the intestinal mucosa into other tissues and organs of the body and the blood circulation [18].

The intestinal barrier is functionally classified into mechanical, chemical, immune, and biological barriers. Specifically, the mechanical barrier is the normal anatomical structure of the intestine, including the mucus layer, intestinal epithelial cells, and the tight junctions between epithelia; the chemical barrier mainly includes gastric acid, various digestive enzymes, and bile; the immune barrier mainly consists of lymphocytes and immunoglobulin A secreted by the intestinal mucosa; the biological barrier consists of the balance of normal flora, which is an important environmental factor for energy absorption and storage. Impairment of intestinal barrier function is mainly manifested by dysbiosis of intestinal flora, excessive growth of small intestinal bacteria, and increased permeability of intestinal mucosa. The intestinal biological barrier maintains a dynamic balance. Experiments in humans [19] showed that the composition of the intestinal flora varied between individuals within a short period of time in response to a change in diet. Normal human intestinal flora ferment undigested food from the digestive organs, increasing the efficiency of energy metabolism and thus providing more energy to the host.

When the balance of intestinal flora is disturbed, the number of conditionally pathogenic bacteria increases and the corresponding normal flora decreases, resulting in impaired energy metabolism. Of course, NAFLD also contributes to the dysbiosis of the intestinal flora. The development of NAFLD is accompanied by the production of various inflammatory mediators. IL-1 and interferon inhibit the feeding centre, reducing appetite and reflexively weakening gastrointestinal motility; prostaglandin 2 and platelet-activating factor cause abnormal intestinal motility, gastrointestinal dysfunction, and reduced or absent migratory motor complexes, with the most important consequence of stagnation of the contents of the small intestine, leading to dysbiosis [20].

The intestinal flora is a complex symbiotic system in the human body, and probiotics can regulate the intestinal microecological balance and play the role of protecting intestinal mucosa, anti-inflammation, and improving lipid metabolism. The dysbiosis of intestinal flora causes acute immune response, and thus, TNF-*α* is expressed in large amounts, which activates the expression of genes with lipid synthesis function, such as SREBP-1c gene fragment, through sensitization, thus promoting hepatocyte steatosis. Probiotics can inhibit the nuclear factor **k**B pathway in intestinal epithelial cells, thereby increasing IL-22 expression, which plays an important role in stabilizing the internal environment and tissue repair and affecting cellular value-added, differentiation, apoptosis, and immune effects by regulating the tyrosine protein kinase-1 (JAK1)/signal transduction-activated transcription factor-3 (STAT3) signaling pathway and downregulating TG synthesis-related genes; the expression of fatty acid transporter protein (FATP) was downregulated to inhibit hepatocyte steatosis. Therefore, probiotics have significant anti-inflammatory and antistatogenic effects and can also reduce TG synthesis [21]. The results of the study showed that probiotic treatment increased serum HMW-APN levels and thus promoted fat metabolism, which is consistent with the findings of Owaga et al. [22]. By anti-inflammatory, promote lipid metabolism and inhibit lipid synthesis, thus restoring liver enzymatic indexes to positive levels, lowering blood lipids, and promoting the improvement of patients' conditions.

There is no ideal drug for the treatment of NAFLD, but recent studies have found that probiotic preparations are effective in the treatment of NAFLD. The therapeutic principle is to use the interaction between the intestine and liver to promote the growth and reproduction of normal microorganisms in order to inhibit the growth of pathogenic bacteria, reduce the production of bacterial endotoxins, inflammatory factors, and other harmful substances, rapidly establish the microecological balance of the gastrointestinal tract and maintain the stability of the intestinal biomucosal barrier. For this reason, more and more physicians tend to use probiotics and other intestinal barrier modulating drugs in clinical practice for the prevention and treatment of NAFLD, but the results are still controversial due to the small number of large-scale clinical studies and ethical issues [23].

## 5. Conclusions

The probiotic preparation used in this study is a live preparation of Bifidobacterium longum, Lactobacillus bulgaricus, and Streptococcus thermophilus. All three form a combined flora that grows under different conditions and has a fast and long-lasting effect.

This study demonstrated that the probiotic preparation improved liver function and dyslipidemia in a healthy population with NADLD and significantly improved hepatocyte steatosis, possibly by regulating the intestinal flora and thereby reducing inflammatory factors and improving insulin resistance. The role of intestinal dysbiosis in the pathogenesis of NAFLD should not be overlooked, and probiotic preparations have many advantages such as less adverse effects and good tolerability, but in terms of the prevention and treatment of fatty liver, its long-term efficacy and the causal relationship with insulin resistance need to be studied more thoroughly.

## Figures and Tables

**Figure 1:** Hepatic steatosis in each group of rats (HE ×400). (a) Control group; (b) model group; (c) treatment group.

**Figure 2:** Infiltration of inflammatory cells in the liver of rats in each group (HE ×400). (a) Control group; (b) model group; (c) treatment group.

**Table 1:** Lipid, liver function, and liver index concentrations in rats (mean ± SD).

Group	*n*	TC (mmol/L)	TG (mmol/L)	ALT (U/L)	AST (U/L)	Liver index
Control group	10	1.72 ± 0.16	0.48 ± 0.09	41.2 ± 0.09	145.8 ± 3.1	2.45 ± 0.24
Model group	12	2.3 ± 0.11	0.90 ± 0.08	88.4 ± 4.3	223.6 ± 4.9	3.78 ± 0.33
Treatment group	12	2.24 ± 0.13	0.52 ± 0.03	55.1 ± 5.9	157.6 ± 2.7	2.58 ± 0.19

Note: the meaning of all abbreviations, group (control, model, and treatment), and the statistical test used.

**Table 2:** Serum inflammatory factor concentrations and insulin resistance index in the healthy group (mean ± SD).

Group	*n*	IL-6 (ng/L)	Adiponectin (*μ*g/L)	TNF-*α* (ng/L)	HOMA-R
Control group	10	0.45 ± 0.18	2.18 ± 0.39	1.92 ± 0.21	5.38 ± 1.12
Model group	12	1.13 ± 0.11	1.42 ± 0.08	2.47 ± 0.13	10.16 ± 0.29
Treatment group	12	0.64 ± 0.13	2.03 ± 0.13	2.09 ± 0.36	6.26 ± 1.23

Note: the meaning of all abbreviations, group (control, model, and treatment), and the statistical test used.

## Data Availability

The experimental data used to support the findings of this study are available from the corresponding author upon request.
